This article has been retracted.

# Effects of Quantitative Nursing Combined with Psychological Intervention in Operating Room on Stress Response, Psychological State, and Prognosis of Patients Undergoing Laparoscopic Endometrial Cancer Surgery

**DOI:** 10.1155/2022/6735100

**Published:** 2022-08-30

**Authors:** Xiaojing Chen, Huiyan Li, Shouyan Wang, Yu Wang, Li Zhang, Dandan Yao, Li Li, Ge Gao

**Affiliations:** ^1^Department of Clean Operation, Harbin Medical University Cancer Hospital, Harbin 150081, China; ^2^Department of Nursing, Harbin Medical University Cancer Hospital, Harbin 150081, China; ^3^Department of Anesthesiology, Harbin Medical University Cancer Hospital, Harbin 150081, China

## Abstract

**Objective:**

To investigate the effects of quantitative nursing and psychological interventions on stress response, mental health, and prognosis in endometrial cancer patients having laparoscopic surgery.

**Methods:**

The random number table approach was used to identify and split 98 patients with endometrial cancer undergoing laparoscopic surgery at our hospital's Obstetrics and Gynecology Hospital (*n* = 49) into observation and control groups (*n* = 49) from May 2020 to February 2022. Both groups received standard care in the operating room, while those in the observation group received quantitative and psychological interventions in the operating room. Both groups were compared for perioperative markers, stress indicators, coping strategies, and pain levels.

**Results:**

In terms of age, TNM stage, or pathology, there was no statistically significant difference between the two groups (*P* > 0.05). Both the observation and control groups experienced statistically significant (*P* < 0.05) reductions in the perioperative markers of operation time, intraoperative blood loss, and overall hospital stay. Both groups' SAS and SDS scores were lower than they had been prior to surgery, but the observation group had lower scores than the control group, and these differences were statistically significant (*P* < 0.05). Postsurgery, the observation group's cortisol and adrenaline levels were lower than those of the control group, and both groups' levels were higher than before surgery, with statistical significance (*P* < 0.05) in both groups. Neither coping style nor pain level differed significantly between the two groups before surgery (*P* > 0.05). Postoperatively, while yield item scores were lower and faces scores were higher than the control group, the observation group's avoidance item score was lower than the control group. All with statistical significance. There were substantial differences in NRS SCORE between observers and controls.

**Conclusion:**

After laparoscopic surgery to remove endometrial cancer, patients may benefit from the combination of quantitative nursing and psychological intervention in the operating room to alleviate postoperative anxiety and sadness and reduce stress reaction.

## 1. Introduction

During the perimenopausal and postmenopausal periods, women are more likely to develop endometrial cancer. It is mainly treated by surgery in clinic [1]. Laparoscopic surgery has the advantages of high safety and less complications during the perioperative period. However, it still causes certain damage to the body. At the same time, due to the impact on the body shape of patients, patients are prone to strong psychological and physical stress reactions, which is not conducive to the work of anesthesiologists and surgeons, leading to poor rehabilitation. Therefore, it is necessary to give patients better medical care and services [2]. The success of the operation, the patient's recovery, and the patient's quality of life after surgery can all be influenced by the quality of the nursing care provided, and the patient's postoperative rehabilitation but conventional nursing cannot meet the above needs and affect the surgical effect to a certain extent, delaying the rehabilitation process [3]. Quantitative nursing in operation room means that through strictly controlling various details and good communication with patients during the whole perioperative period, risks caused by insufficient preparation are avoided, which can effectively remedy the disadvantages of conventional nursing in operation room and quantify the nursing scheme in operation room, thus ensuring the smooth operation and safety of patients [4]. Although relevant studies in China and overseas have demonstrated that psychological counseling can successfully improve patients' physical and mental status, the influence on whether stress response is improved is still unclear [5]. In 98 patients who underwent laparoscopic surgery for endometrial cancer and were admitted to the Department of Obstetrics and Gynecology Hospital at our hospital from May 2020 to February 2022, the stress response and psychological state of our patients were compared and observed following various nursing interventions. The following are the outcomes of the study.

## 2. Material and Methods

### 2.1. General Material

Using the random number table, 98 patients who underwent laparoscopic surgery for endometrial cancer at our hospital between May 2020 and February 2022 were chosen as research participants and split into two groups: an observation group (*n* = 49) and a control group (*n* = 49). In the observation group, quantitative nursing in the operating room was paired with psychological intervention, and the control group received standard intervention, however. The participant in this experiment gave informed consent, which was authorized by a hospital's Ethics Committee.

### 2.2. Criteria of Inclusion and Exclusion

Inclusion criteria [6] are (1) endometrial cancer is diagnosed according to clinical manifestations and auxiliary examinations such as imaging, (2) tolerant to surgery, (3) the I–II scale set by the American Association of Anesthesiologists, (4) no surgery or hemorrhagic disease within six months, and (5) informed consent forms are signed by patients and their families.

Exclusion criteria [7] are (1) tumor metastasis has occurred, (2) together with other cancerous tumors, (3) combination of cardiovascular and cerebrovascular illness, (4) liver and kidney dysfunction, and (5) confusion or cognitive impairment.

### 2.3. Nursing Methods

Treatment was kept to a minimum for those in the control group. The preoperative diet guidance, explain the complications; Active cooperation with doctors and nurses during the operation and strict monitoring of patients' vital signs; Postoperative guidance on the correct medication and discharge guidance, etc. Quantitative nursing in operation room is combined with psychological intervention for patients in observation group. Specific measures are as follows:

1. *Presurgery Quantification*. The age, disease status, and combined disease status of patients were obtained. (1) In terms of age, one point before the age of 50, two points from 50 to 60, and three points above the age of 60 are counted. (2) There were 10 items on the SAS and SDS scales, which both used the four-grade scoring approach, and disease quantification was assessed using the SAS and SDS scales. The total scores were 100 points. A lower score indicated a milder anxiety or depression. Mild anxiety or depression 50–60 points were scored as one point, moderate anxiety or depression 61–70 points were scored as two points and >70 points were scored as three points. (3) Quantification of combined diseases: 1 point without complications, 2 points with one disease, and 3 points with more than two diseases. (4) The total scores of low-risk nursing patients undergoing surgery were <4 points, with medium-risk of 4–6 points and high-risk of >6 points. The grades were N1, N2, and N3 according to the nurse's title, seniority, and nursing skills. Patients with low risk of surgery, equipped with N1 level nurses, nurse-patient ratio of 1 : 2. Patients at risk during the operation were equipped with N2-level nurses, and the ratio of nurses to patients was 1 : 1. High-risk patients undergoing surgery were equipped with N3-level nurses, and the nurse-patient ratio was 2 : 1. During the implementation, the nurses were evaluated and adjusted according to the timely feedback information
2. *Preoperative Cognitive Intervention*. Knowledge seminars and health handbooks were used to explain the disease-related knowledge and treatment plan to the patients. The medical staff explained the possible discomfort during the operation and the possible complications after operation to the patient with the help of videos and pictures and issued the certificate, with emphasis on the effect of the operation on his physiological function. Spouse is an important participant in patient education. While educating and educating patients, medical staff explained the care methods and related knowledge of female reproductive system to the spouse, in order to reduce the psychological burden of the patient's spouse and encourage them to care for the patient
3. *Intraoperative Care*. Cooperate with the surgeon in skin preparation, posture placement, device link, and pipeline examination, and cooperate with the anesthesiologist in the anesthesia, ventilator, and other device examinations. Patients' vital signs were closely observed during the operation, and the parameters of various instruments were adjusted timely according to needs. After the operation, cooperate with the doctor for instrument inspection, assist the doctor for disinfection and incision suture, etc. Meanwhile, the mental state and vital signs of the patients after anesthesia and sobriety were observed
4. *Postoperative Care*. Cooperate with the doctor to check the placement of drainage tube and drainage, and record the pain of the patients as well as the use of analgesic pump after operation. The postoperative precautions were informed, and the patients were advised to choose their favorite exercise mode and take reasonable exercise every day to enhance physical strength. The exercise time was controlled at 20 min, and it was conducted twice a day
5. *Psychological Intervention*. Nursing staff chose an appropriate time every day to communicate with the patients and their families to understand the root causes of negative emotions in patients. It was shown that hypnosis, image dialogue therapy, cognitive therapy, and other methods were effective in helping patients destress and unwind in order to alleviate symptoms of stress, such as anxiety and depression. As well as being educated on how their emotional state affects the treatment of sickness, so that they could understand that the good or bad mood directly affected the prognosis and subsequent treatment. In addition, patients are taught some psychological adjustment methods to guide relaxation training and to enter a relaxed state consciously by feeling the difference between muscle tension and relaxation. Medical staff organized patients with similar symptoms to participate in the communication meeting so as to encourage and help each other and give full play to the peer effect. During this period, medical staff also need to do a good job in the ideological work of their families, to guide them to play their due role of supervision and accompanying them, to affect the patients with their own optimistic state, and to enable the patients to deal with the treatment in a positive attitude

### 2.4. Serum Test

All patients collected 5 mL of venous blood in the morning on an empty stomach and allowed to stand at room temperature for half an hour. When serum appeared in their layers, they were placed in a centrifuge, and the upper layer of serum was sucked after centrifuging at a speed of 3000 r/min for 10 minutes. The test samples were stored in a refrigerator at −80°C. Cortisol was determined by radioimmunoassay, and epinephrine was determined by immunofluorescence assay.

### 2.5. Observational Index

1. In terms of perioperative indicators, the two groups were compared in terms of operation time, intraoperative bleeding volume, and hospital stay
2. The stress levels of the two groups were evaluated before and 24 hours after the operation. Psychological and physical indicators are also included. Cortisol and epinephrine levels were measured using the SAS and SDS scores to examine psychological and physiological signs
3. A comparison of the two groups' coping styles before and 24 hours after surgery was made. Medical coping model questionnaire (MCMQ) was used. The questionnaire consisted of three dimensions of avoidance (7 items), submission (6 items), and facing (7 items), with a total of 20 items. Each item adopted a 4-level scoring system, which represented that it had never been like this, sometimes like this, often like this, and always like this. The higher score indicated that patients were more inclined to the coping style of this item
4. Prior to and 24 hours after surgery, both groups were tested for pain levels. Each patient's level of pain was evaluated using the numerical rating scale (NRS), with 0 denoting no pain at all and 10 denoting the most painful and extreme agony

### 2.6. Statistical Analysis

SPSS22.0 statistical software was used to conduct the analysis. They employed the *t*-test to compare the groups based on the mean standard deviation of the measurement data ($\overset{®}{x}\pm s$). The percentage (percent) and number (*N*) of enumeration data were compared using the *χ*^2^ test. The difference was deemed statistically significant at <0.05.

## 3. Results

### 3.1. General Material

As indicated in Table 1, there was no significant difference between the two groups in terms of age, TNM stage, and pathological type (*P* > 0.05).

### 3.2. Perioperative Indicators of Patients

There was a statistically significant difference (*P* < 0.05) in perioperative markers such operation duration, intraoperative bleeding volume, and total hospital stay between the observation group and the control group, as shown in Table 2 and Figure 1.

### 3.3. Stress Indicators of Patients

Following surgery, patients' SAS and SDS ratings were lower in both groups than they were before to surgery, as indicated in Table 3, the observation group's scores were lower than the control group, which had a statistically significant difference (*P* < 0.05). In terms of physiological indicators, the postoperative observation group's cortisol and epinephrine levels were lower than those in the control group, and the postoperative two groups' levels were higher than those prior to surgery in the two postoperative groups. *P* < 0.05 was the threshold for statistical significance in this study, as shown in Table 3 and Figure 2.

### 3.4. Two Groups of Patients' Coping Styles

Before surgery, there were no significant differences in the two groups' coping methods (*P* > 0.05). The avoidance and yielding item scores of the observation group were lower than those of the control group, however, the facing item scores of the observation group were higher than those of the control group.  Table 4 and Figure 3 show that the differences were statistically significant. Cores are between the observation and control groups.

### 3.5. Pain Severity in Two Groups

Both groups saw no significant differences in discomfort prior to surgery (*P* > 0.05).  Table 5 and Figure 4 show that after the operation, there was a statistically significant (*P* < 0.05) difference in NRS scores between the observation and control groups.

## 4. Discussion

At present, for patients with early endometrial cancer clinically, surgical resection is generally adopted to avoid the lesions from further development. There are numerous advantages to laparoscopic surgery, including reduced trauma. However, since the operation involved reproductive organs, and the patients' immune function was lower than that of the healthy ones, there was a certain operation risk. At this time, bad emotions and body damage would easily induce stress response in the body [8]. Excessive stress response will destroy the endocrine and nervous system balance of patients, affecting the surgical effect and subsequent rehabilitation. Obviously, simple routine care can no longer solve such problems.

Studies have shown that developing targeted care programs based on patients' disease characteristics can reduce patients' anxiety and depression during the operation and urge patients to actively cooperate with medical work during the operation [9]. Quantitative nursing in operation rooms is a brand-new clinical nursing mode, in which the nursing plan is reasonably formulated based on the patient state, standardized, and quantified evaluation and classification, as a means to improve the overall prognosis of the patient by increasing their participation with surgery and decreasing their perioperative trauma psychologically and physiologically [10]. For patients undergoing laparoscopic surgery to remove uterine fibroids, clinical trials have indicated that a nursing intervention in the operating room improves both the surgical outcomes and the patients' emotional well-being. Other studies have demonstrated that psychological assistance in patients having laparoscopic resection can improve their psychological condition and stabilize their vital signs [11, 12].

According to the findings of this study, the observation group's perioperative indicators, such as operating time, the amount of blood lost during surgery, and the length of time the patient spent in the hospital, were both less than in the control group. It has been found that endometrial cancer patients who got quantitative nursing during surgery in addition to psychological assistance recovered more quickly. It was analyzed that in the present study, nurses with different qualifications and nursing skills were assigned to patients of different grades through quantitative classification of age, disease status, and combined diseases of endometrial cancer patients; and targeted intervention [13] was conducted to enable patients to receive treatment with an understanding of endometrial cancer and the process of laparotomy, ensure that patients with different psychological states and conditions can receive professional care, eliminate fear of diseases and surgery, and enhance confidence in coping with the discomfort caused by surgical trauma, so that they can actively receive treatment, improve the treatment effect, and promote the stable improvement of the condition [14].

According to reports, when the mental state of the human body is in extreme conditions, such as anxiety, depression, or excessive tension, the sympathetic nerve will be overexcited, causing the release of excessive catecholamine, promoting the increase of cortisol and epinephrine levels, and resulting in the excessive increase or decrease of heart rate and blood pressure [15, 16]. It has been noted that psychological intervention may be able to lower the body's stress reaction by inhibiting the natural defense system's increase in adrenocortical hormone. Both groups' SAS and SDS scores were lower after surgery than they were before, but the observation group's scores were lower than those of the control group, and the differences were statistically significant. All three groups had higher levels of cortisol and epinephrine after surgery than before, indicating that they had been exposed to more stress than their presurgical counterparts. Statistically significant differences were found. Patients undergoing laparoscopic surgery for endometrial cancer could benefit from quantitative nursing in the operating room, as well as psychosocial counseling, according to the study. The analysis showed that some extreme emotions such as fear and anxiety were avoided through popularization of disease-related knowledge, correction of patients' wrong cognition, and establishment of correct concept of treatment during nursing [17]. In addition, psychological counseling is conducted for the patients to achieve the optimal psychological state as much as possible so as to regulate the hypothalamic and adrenal sympathetic nervous system of the patients and reduce the massive secretion of cortisol and adrenocortical hormone in the body caused by negative emotions, thereby avoiding stress response to a great extent [18].

Research has shown that when patients develop fear of death due to lack of understanding of cancer, they are prone to develop cancer-related fatigue and adopt such methods as “avoiding” and “yielding” to cope with the disease. The above two coping methods not only aggravate the negative emotions of patients but also lead to physiological discomforts such as pain, aggravate the development of the disease, and lead to the decline of patients' life quality [19]. A lower avoidance and yield item score in the observation group after surgery, as well as a significantly higher face item score, was seen in comparison to the control group. Endometrial cancer patients who received quantitative nursing in the operating room as well as psychological assistance improved their coping methods following laparoscopic surgery, according to these findings. The analysis suggests that the quantitative nursing in operation room combined with psychological intervention can promote the patients to affirm their life values and stimulate their positive potentials [20] by improving their treatment concepts and giving them the confidence to fight against diseases and face treatment actively with the help of spouse's encouragement and family support, thus alleviating the loneliness caused by illness and enabling patients to correctly treat the physiological reactions caused by diseases with an optimistic attitude, thus avoiding the states of avoidance and submission, and thus becoming stronger [21].

The experimental group's postoperative NRS scores were much lower than those of the controls, despite the fact that preoperative pain levels did not differ significantly between the two groups, and this difference was statistically significant. Preoperative pain levels did not change substantially between the two groups; however, postoperative NRS scores were markedly lower in the experimental group compared to controls, indicating a meaningful effect of surgery. It was analyzed that quantitative nursing in operation room combined with psychological intervention helped patients to be willing to face the disease directly, and the state of patients at this time was extremely beneficial to the implementation of various medical operations, equivalent to improving their treatment compliance, and beneficial to transferring patients' attention to pain and reducing their pain perception [22]. In addition, after the patients have a certain understanding of disease management, some wrong behavior patterns can be avoided as far as possible to greatly reduce the generation of additional pain, wherein the prognosis is much enhanced [23, 24].

The combination of quantitative nursing and social psychological intervention in operating room is a new nursing model that appears with the rapid development of psychology. It affects the psychological state of patients through various nursing and psychological means, so as to achieve the purpose of creating a good psychological environment for treatment and rehabilitation for patients. The research results show that the team nursing after the SAS and SDS scores was lower than the control group, indicating that the operating room quantitative nursing combined with social psychological intervention can effectively relieve patients with endometrial cancer perioperative anxiety and depression, and the quantitative results show the operating room nursing combined with social psychological intervention to improve the patients quality of life also have certain help, this is for In psychological care is also a kind of comprehensive care, its targeted psychological counseling to patients at the same time, also other factors that is likely to affect the psychological status of patients with nursing intervention, so as to reduce the patients fear of the unknown, to guide the patient is distracting to avoid overly concerned about their disease patients, and families with help to urge patients to feel from the family Care. This study also has obvious clinical application value. However, the sample size of this study is small, and the survival rate of patients has not been determined, so the results have certain limitations, and it is necessary to further accumulate the sample size to conduct in-depth research.

## Figures and Tables

**Figure 1:** Perioperative indicators of patients between the two groups. Compared with control group, ^∗^*P* < 0.05, the differences were statistically significant.

**Figure 2:** Patients' coping styles between the two groups. Compared with control group, ^∗^*P* < 0.05, the differences were statistically significant.

**Figure 3:** Patients' coping styles between the two groups. Compared with control group, ^∗^*P* < 0.05, the differences were statistically significant.

**Figure 4:** Pain levels between the two groups. Compared with control group, ^∗^*P* < 0.05, the differences were statistically significant.

**Table 1:** Comparison of the general material between the two groups.

Group	Control group	Observation group	Total value	*P* value
Age (years, $\overset{®}{x}\pm s$)	52.54 ± 10.72	52.12 ± 10.68	1.252	0.062
TNM grade (cases, *n*)				
Grade II	27	28	0.874	0.312
Grade III	22	21		
Pathological type (cases, *n*)				
Endometrioid adenocarcinoma	23	24	0.754	0.385
Adenosquamous carcinoma	17	19		
Clear cell carcinoma	9	6		

**Table 2:** Comparison of perioperative indicators of patients between the two groups ($\overset{®}{x}\pm s$).

	Control	Observation
Operative time (min)	188 ± 11.74	145 ± 9.52
Intraoperative blood loss (ml)	321 ± 23.01	245 ± 18.45
Total length of hospital stay (d)	10.33 ± 2.97	7.35 ± 1.13

**Table 3:** Comparison of patients' coping styles between the two groups ($\overset{®}{x}\pm s$).

	Control	Observation
SAS		
Before	61.45 ± 9.88	61.47 ± 9.13
After	42.31 ± 7.56	32.78 ± 5.20
SDS		
Before	51.51 ± 8.20	51.53 ± 7.98
After	45.26 ± 7.31	28.66 ± 2.19
Cortisol, ng/L		
Before	101.23 ± 10.11	101.16 ± 11.63
After	140.89 ± 20.17	120.36 ± 15.08
Drenaline, ng/L		
Before	90.15 ± 8.75	90.12 ± 8.34
After	150.05 ± 21.53	128.88 ± 16.89

**Table 4:** Comparison of patients' coping styles between the two groups ($\overset{®}{x}\pm s$).

	Control	Observation
Duck		
Before	25.21 ± 3.78	24.96 ± 3.83
After	19.53 ± 3.06	7.53 ± 1.10
Yield		
Before	24.1 ± 3.75	23.64 ± 3.96
After	18.53 ± 3.51	7.83 ± 1.09
Face		
Before	7.03 ± 1.07	6.98 ± 1.01
After	9.36 ± 1.09	15.73 ± 2.74

**Table 5:** Comparison of pain levels between the two groups ($\overset{®}{x}\pm s$).

Group		Control	Observation
NRS	Before	6.29 ± 1.12	6.36 ± 1.04
	After	4.52 ± 1.01	2.18 ± 0.43

## Data Availability

The data used to support the findings of this study are available from the corresponding author upon request.
